The article "Clinical Efficacy of LSC and TVT-O for Stress Urinary Incontinence Complicated with Pelvic Organ Prolapse and Factors Influencing Postoperative Urinary Function Recovery" was retracted in 2023. Reasons: suspected computer-generated content; unreliable results or conclusions; concerns about the data; concerns about the results or conclusions.

# Clinical Efficacy of LSC and TVT-O for Stress Urinary Incontinence Complicated with Pelvic Organ Prolapse and Factors Influencing Postoperative Urinary Function Recovery

**DOI:** 10.1155/2022/1557256

**Published:** 2022-03-07

**Authors:** Wenling Du, Zhihu Liu, Daya Wang

**Affiliations:** ^1^Department of Gynecology and Obstetrics, Wenzhou Central Hospital, Wenzhou 325000, Zhejiang, China; ^2^Department of Urology, Beidahuang Industry Group General Hospital, Harbin 150088, Heilongjiang, China; ^3^Department of Urology, Wenzhou Central Hospital, Wenzhou 325000, Zhejiang, China

## Abstract

Pelvic organ prolapse is caused by various causes, which leads to the weakness of the tissue supporting the pelvic floor and then causes the downward displacement of female reproductive organs and adjacent organs. Clinical studies have shown that pop is often associated with stress urinary incontinence. This research project aimed to clarify the clinical effect of laparoscopic sacrocolpopexy (LSC) and tension-free vaginal tape obturator (TVT-O) for stress urinary incontinence (SUI) complicated with pelvic organ prolapse (POP) and the influencing factors of postoperative urinary function (UF) recovery. The clinical data of 125 patients with SUI complicated with POP treated in Wenzhou Central Hospital and Beidahuang Industry Group General Hospital between March 2018 and December 2019 were retrospectively analyzed. Patients were assigned to the following two arms based on different treatment methods: the combination group (*n* = 65, treated with LSC plus TVT-O) and the control group (*n* = 60, treated with LSC). The alterations of perioperative clinical and urodynamic indexes were analyzed. The objective and subjective response rates were observed and compared. The degree of POP before and after surgery was evaluated. According to the urinary function recovery time, the patients were divided into the fast and non-fast recovery groups, and then, the factors influencing postoperative UF recovery were analyzed between groups. The combination group showed statistically longer operation time (OT) and postoperative indwelling catheter and higher intraoperative blood loss (IBL) than the control group (all *P* < 0.05), but the anal exhaust time and postoperative length of stay (LOS) differed insignificantly between the two arms. The combination group outperformed the control group in the objective response rate, as well as the scores of illness, quality of life (QOL), and sexual life (all *P* < 0.05). Menopause, maximum flow rate (MFR), and preoperative residual urine volume were identified as the influencing factors for normal urination. For patients with SUI complicated with POP, the efficacy of laparoscopic sacrocolpopexy was limited, while combining with TVT-O would obtain more significant short-term and long-term efficacy, which can significantly improve patients' urination and long-term quality of life, with higher safety and clinical promotion value.

The article "Clinical Efficacy of LSC and TVT-O for Stress Urinary Incontinence Complicated with Pelvic Organ Prolapse and Factors Influencing Postoperative Urinary Function Recovery" was retracted in 2023. Reasons: suspected computer-generated content; unreliable results or conclusions; concerns about the data; concerns about the results or conclusions.

## 1. Introduction

Pelvic organ prolapse (POP) and stress urinary incontinence (SUI) both fall into the category of pelvic floor diseases that seriously compromise women's quality of life (QOL) [1]. POP, a commonly seen pelvic floor tissue disease, is the primary presentation of pelvic floor dysfunction including swelling or prolapse of pelvic organs such as vagina, bladder, uterus, and rectum, manifesting as discomfort such as changes in urination and defecation [2, 3]. SUI, on the other hand, refers to “the chief complaint of involuntary uracratia due to exertion or physical activity, or sneezing or coughing” [4]. The global prevalence of POP and urinary incontinence was 19.7% (range 3.4–56.4%) and 28.7% (range 5.2–70.8%), respectively [5]. Clinical evidence has shown that POP, associated with SUI, has a predilection for middle-aged and elderly women [6]. Marschke et al. [7] reported that the risk of POP and recurrence increases with age and changes in menstrual status. In China, the prevalence of POP grows steadily with the increasingly severe population aging, with approximately one fifth of women needing surgical treatment for SUI or POP in their lifetime, according to statistics [8]. Hysterectomy is the mainstay of early treatment for POP, but this approach is prone to cause vaginal vault prolapse, resulting in iatrogenic injury [9]. Moreover, the lifetime surgical risk of POP is 13%, and up to 17% will undergo reoperation [10, 11]. For patients with SUI, the midurethral sling is a minimally invasive surgical technique for the treatment of Sui. The symptom cure rate is 75–94%, and the objective cure rate is 57–92% [12]. However, for those with POP and SUI, whether to simultaneously perform anti-SUI surgery in the treatment of POP is still controversial given the few domestic and foreign research on this issue.

Since the introduction of the integral theory of pelvic floor in 1990, artificial pelvic repair has been widely used and recognized in clinic, with encouraging results [13]. As the minimally invasive technology advances, laparoscopic sacrocolpopexy (LSC) has gradually replaced transabdominal surgery in virtue of its clear surgical vision, less trauma, less bleeding, and faster postoperative recovery and is currently recognized to be the golden criterion for apical prolapse treatment [14]. Midurethral sling surgery, such as tension-free vaginal tape and tension-free vaginal tape obturator (TVT-O, also known as trans-obturator suburethral tape from inside to outside), is the surgical modality most extensively applied to treat SUI with urethral hypermobility [15]. Midurethral sling surgery is the most widely studied surgical treatment method with a high safety profile for female SUI. The sling contributes to good short- and medium-term results, irrespective of the method of insertion [16]. In recent years, there have been reports on LSC for patients with POP [17]. However, little research has discussed TVT-O application in POP procedure, and there is a lack of follow-up and evaluation of patients' postoperative QOL. Accordingly, we retrospectively analyzed the clinical effect of LSC combined with TVT-O in POP patients complicated with SUI in Wenzhou Central Hospital and Beidahuang Industry Group General Hospital and conducted medium- and long-term follow-up on patients. Our selection criteria include surgical operations for POP with or without continence procedures in continent or incontinent women. Our primary outcome was subjective postoperative POP, and secondary outcomes included urodynamic condition, postoperative complications, and voiding dysfunction, to further comprehensively evaluate the clinical value of the two procedures, to provide more convincing evidence for the selection of specific clinical treatment plan.

The article "Clinical Efficacy of LSC and TVT-O for Stress Urinary Incontinence Complicated with Pelvic Organ Prolapse and Factors Influencing Postoperative Urinary Function Recovery" was retracted in 2023. Reasons: suspected computer-generated content; unreliable results or conclusions; concerns about the data; concerns about the results or conclusions.

## 2. Materials and Methods

### 2.1. Participants

125 patients with SUI complicated with POP treated in Wenzhou Central Hospital and Beidahuang Industry Group General Hospital between March 2018 and December 2019 were collected and analyzed retrospectively. They underwent LSC or TVT-O in our department. The choice of surgical procedure is initially based on the patient's willingness to undergo surgery and the specific circumstances of each patient.

Patients were assigned to the control group (accepted LSC, *n* = 60) and the combination group (accepted LSC combined with TVT-O, *n* = 65) according to different treatment methods. The study followed the ethics standards for clinical trials, and the Medical Ethics Committee of Wenzhou Central Hospital and Beidahuang Industry Group General Hospital approved the study protocol (No. 202111041455000544727).

Inclusion criteria are as follows: those with vaginal vault, anterior vaginal wall, and/or uterus prolapse (II-IV degree) according to the Pelvic Organ Prolapse Quantification (POP-Q) system [18]; SUI confirmed by the International Consultation on Incontinence Questionnaire-Short Form (ICIQ-SF) [19]; and positive Marshall-Bonney and tension test results. The degree of SUI was graded by the Ingelman-Sundberg Classification; patients who received surgical treatment; patients who were successfully followed up, with complete clinical data; and those who gave informed consent to the study and cooperated with the data collection work. Exclusion criteria are as follows: coagulation dysfunction; urinary incontinence (UI) due to urge UI and filling UI; overactive bladder and bladder emptying disorders; severe heart, lung, liver, and kidney dysfunction; and incomplete follow-up data. The general baseline data were similar in the two arms (*P* < 0.05), suggesting comparability Table 1.

The article "Clinical Efficacy of LSC and TVT-O for Stress Urinary Incontinence Complicated with Pelvic Organ Prolapse and Factors Influencing Postoperative Urinary Function Recovery" was retracted in 2023. Reasons: suspected computer-generated content; unreliable results or conclusions; concerns about the data; concerns about the results or conclusions.

### 2.2. Methods

All patients or their families were informed in detail about the risks of the operation. Three days before surgery, all patients were treated with potassium permanganate diluted sitz bath and iodophor vaginal scrubbing to confirm that there were no other ulcer symptoms in the vagina. Preoperative vaginal douche, skin preparation, and enema were performed, and intraoperative prophylactic antibiotics were given intravenously.

The control group received LSC: all the operations were completed by the same chief physician. The anesthesia was performed by endotracheally intubated intravenous combined anesthesia, and fentanyl 0.1 mg, propofol 100 mg, and succinylcholine 100 mg were used for rapid induction and tracheal intubation followed by universal anesthesia machine to control breathing. During the operation, atracurium and fentanyl were injected intermittently, and propofol was maintained at 6–8 mg/kg·h. In the lithotomy position, the patient had the head low and hip high, and the left low and right high, so that the sigmoid colon was slightly inclined to the left rear. The right and inferior platform area of the sacral promontory was exposed under the laparoscope, avoiding the right ureter. Then, the anterior sacral promontory peritoneum was opened longitudinally from 1.0 cm above the sacral promontory with an ultrasound knife to expose the presacral area, and the lateral peritoneum was opened to the vaginal vault along the medial side of the right uterosacral ligament. Vaginal hysterectomy was performed according to the conventional method. After separating the vesicovaginal space from the rectovaginal space, the mesh (GYNECARE GYNEMESH™ PS, polypropylene mesh, Johnson & Johnson Company, USA) was cut into anterior and posterior lobes. The vaginal segment of the anterior lobe was 3.50 cm × 3.50 cm, which was placed in the paravaginal-paravesical space, and the abdominal segment was 3.00 cm × 11.00 cm; the mesh size of the posterior lobe was 3.00 cm × 15.00 cm, of which 3.00 cm × 3.00 cm was placed in the paravaginal-pararectal space. Using braided absorbable suture 2.0 sutures, the mesh was fixed with 9 stitches intermittently. After disinfection, the mesh was sent into the abdominal cavity via the vagina, and the vaginal stump was sutured. The lens was placed into the abdomen again, and the mesh was pulled and unfolded under the laparoscope. Thereafter, the mesh, which was sutured and fastened to the first sacral vertebra's anterior longitudinal ligament to make sure that the C point was above −6 cm, was then embedded in the retroperitoneum with absorbable lines. Finally, the vagina was filled with iodophor gauze.

The article "Clinical Efficacy of LSC and TVT-O for Stress Urinary Incontinence Complicated with Pelvic Organ Prolapse and Factors Influencing Postoperative Urinary Function Recovery" was retracted in 2023. Reasons: suspected computer-generated content; unreliable results or conclusions; concerns about the data; concerns about the results or conclusions.

Patients in the combination group received LSC combined with TVT-O performed by the same chief physician. TVT-O was performed after LSC. An incision of about 0.5 cm was made at the junction of the patient's clitoris and inner thigh skin folds to separate the bladder space and vaginal mucosa, and the position between the anterior wall of the vagina and the hypourethral groove was cut along the midline until the obturator membrane, with a length of about 2 cm. Then, the puncture needle with mesh was lifted from the submucosa of the right vaginal incision edge and pierced through the avascular area in the right obturator foramen (2 cm adjacent to the clitoris). The operation was completed on the left side in the same way. After adjusting the length of the sling, the plastic cover of the sling was removed and the redundant sling was cut off. Finally, the wound was cleaned carefully, the vaginal mucosa was sutured conventionally, and the gauze was inserted.

All patients had routine antibiotics to fight infection after surgery, and the vaginal gauze was removed timely. Residual urine volume (RUV) was measured by ultrasound, with less than 100 mL considered normal. In case that the RUV was over 100 mL, the catheter or indwelling was extubated as appropriate until reaching the standard. Patients were instructed not to do heavy physical labor within 8 weeks and not to have sex within 12 weeks.

### 2.3. Clinical Data Collection

1. Perioperative evaluation indexes: the operation time (OT), intraoperative blood loss (IBL), length of stay (LOS), and postoperative indwelling catheter time and exhaust time were compared.
2. Postoperative urodynamics: the postoperative urodynamics of the two groups, mainly assessed from initial bladder volume, maximum bladder volume, maximum flow rate (MFR), and recovery time of urinary function (UF), were compared between the two arms.
3. Postoperative complications: complications (defecation discomfort, infection, dysuria, and bladder injury) were observed in both arms.
4. Evaluation of objective response rate (ORR): before and 6 months postsurgery, patients were assessed by the POP-Q system for the degree of POP. Patients were urged to empty their bladder and rectum as much as possible prior to examination or perform Valsalva maneuver and cough during examination to maximum the prolapse of pelvic organs. Vaginal examination and POP-Q were performed to evaluate the objective cure rate. During examination, the efficacy of POP-Q was evaluated by measuring two anatomical points Aa and Ba on the top of vagina and on anterior and posterior walls, Ap and Bp points on the posterior wall, C and D points at the apex, and the total vaginal length (TVL). Within 6 months after surgery, the POP-Q score greater than 0 and less than II indicated that the surgery was successful, and ≥II indicated that the surgery had failed. A score of ≥II six months after surgery indicated recurrence. Cure referred to complete disappearance of symptoms, improvement was considered partial disappearance of symptoms, and ineffectiveness corresponded to non-disappearance of symptoms.
5. Evaluation of subjective response rate: according to patients' medical records and their description, the questionnaires were completed during the preoperative and one-year follow-up after surgery. The questionnaires used in this study included the following: the Pelvic Floor Distress Inventory Short-Form 20 (PFDI-20), with 20 items in total, was adopted for investigating the condition of patients, assessing the impact of the disease on patients' QOL, bowel prolapse, urination-related symptoms, etc., with 0–4 points for each item and 0–80 points for the total score. The higher the score, the worse the patient's recovery. The QOL assessment adopted the Pelvic Floor Impact Questionnaire Short-Form 7 (PFIQ-7) [20]: involving 7 questions, and the questionnaire has 21 items in total (each item: 0–4 points, total score: 0–84 points). The score was inversely proportional to the patient's QOL. Patients were also evaluated for sexual life quality using the Pelvic Organ Prolapse Sexual Questionnaire Short-Form 12 (PISQ-12) [21]: the questionnaire involved 12 questions, with each item scoring 0–4 points and the total score 0–48 points. Higher scores were associated with better sexual life quality.

The article "Clinical Efficacy of LSC and TVT-O for Stress Urinary Incontinence Complicated with Pelvic Organ Prolapse and Factors Influencing Postoperative Urinary Function Recovery" was retracted in 2023. Reasons: suspected computer-generated content; unreliable results or conclusions; concerns about the data; concerns about the results or conclusions.

### 2.4. Statistical Methods

The data from a preliminary study suggest a study power of 80% (*α* = 0.05, *β* = 0.2). Assuming 90% effective rate in the combination group and 70% effective rate in the control group, the sample size required for each arm should be 59, with 118 in total for adequate data acquisition (PASS 15.0, NCSS Statistical Software, Kaysville, Utah).

The statistical software used in this study was SPSS 21.0 (IBM, Armonk, NY, USA) Counting data (*n* (%)) were compared by the chi-square test. The independent-samples t-test was employed to identify the difference in measurement data conforming to normal distribution, which were given (mean ± SD), while the one-way ANOVA and the Bonferroni post hoc analysis were carried out for multigroup comparisons, with *α* = 0.05 as the test standard, and the difference level was set at *P* < 0.05.

## 3. Results

### 3.1. Perioperative Evaluation Indexes

The combination group showed statistically longer OT and postoperative indwelling catheter time and higher IBL than the control group (*P* < 0.05), whereas the two arms showed no evident difference in terms of anal exhaust time and postoperative LOS (*P* > 0.05) (Table 2).

### 3.2. Urodynamic Examination of Patients

The RUV differed insignificantly between the combination group and the control group before surgery (*P* > 0.05). Postoperatively, the control group outperformed the combination group in the initial bladder volume, maximum bladder volume, MFR, and average UF recovery time (*P* < 0.05). The UF recovery time less than or equal to 3 days was considered as rapid recovery, and that more than 3 days was considered as non-rapid recovery. In the control group, 10 cases recovered quickly and 50 did not recover quickly, while in the combination group, 24 cases recovered quickly and 41 cases did not recover quickly. The UF recovery differed statistically between the two arms (*P* < 0.05) (Table 3).

### 3.3. POP-Q Parameter Measurement at Each Reference Point

Compared with those before surgery, the reference points Aa, Ba, Ap, Bp, C, and D improved evidently in both arms at 6 months postoperatively (*P* < 0.05), whereas the intergroup comparison revealed no distinct difference in points Aa, Ba, Ap, and Bp between the control and combination groups (*P* > 0.05), while obvious differences in points C and D at 6 months postoperatively (*P* < 0.05). The intragroup comparison revealed no obvious difference in TVL in the control group before surgery and half a year postsurgery (*P* > 0.05); however, the TVL in the combination group increased markedly half a year postsurgery and was notably longer compared with the control group (*P* < 0.05) (Table 4).

### 3.4. ORR

The cure rate, improvement rate, ineffective rate, and recurrence rate in the control group were 58.3%, 25.0%, 10.0%, and 6.7%, respectively, while those in the combination group were 84.6%, 10.8%, 4.6%, and 0, respectively. The ORR was significantly better in the combination group versus the control group (*P* < 0.05) (Table 5).

### 3.5. Patients' Condition, QOL, and Sexual Life

Preoperatively, there was no distinct difference in PFDI-20, PFIQ-7, and PISQ-12 scores between the combination and control groups (*P* > 0.05). One year after surgery, two groups all showed markedly lower PFDI-20 and PFIQ-7 scores and higher PISQ-12 score, and the degree of change is more significant in the combination group than in the control group (*P* < 0.05) (Figure 1).

The article "Clinical Efficacy of LSC and TVT-O for Stress Urinary Incontinence Complicated with Pelvic Organ Prolapse and Factors Influencing Postoperative Urinary Function Recovery" was retracted in 2023. Reasons: suspected computer-generated content; unreliable results or conclusions; concerns about the data; concerns about the results or conclusions.

### 3.6. Incidence of Complications

Defecation discomfort, infection, dysuria, and bladder injury were observed in 1, 1, 2, and 0 cases, respectively, in the combination group, while those were found in 2, 3, 3, and 3 cases, respectively, in the control group. The complication rate was notably higher in the control group versus the combination group (18.3% *vs* 6.1%, *P* < 0.05) (Table 6).

### 3.7. Influencing Factors of Postoperative Urination Recovery

According to the results in Table 3, among all patients, the recovery time of urination was rapid in 34 cases and non-rapid in 91 cases. Age, menopause, underlying diseases, MFR, and preoperative RUV were observed in relation to the recovery time of urination. The results showed that menopause, MFR, and preoperative RUV were associated with normal micturition (*P* < 0.05), while age and underlying diseases were not (*P* > 0.05) (Table 7).

## 4. Discussion

Female pelvic structure is mainly composed of bones, muscles, ligaments, and organs [22]. Petros and Ulmsten [13] believe that the female pelvic floor is a multipart organic whole, and the damage of the pelvic floor structure will lead to its abnormal shape and function, which can be restored to a certain extent through structural repair. Theoretically, artificial repair can improve or even cure pelvic floor dysfunction. In addition, relevant studies suggest that POP and SUI have similar etiology and pathogenesis, and the two often coexist [23, 24]. Therefore, concurrent anti-SUI is the key to treating POP. The treatment of POP with or without SUI depends on the severity of prolapse, related symptoms, women's wishes and general health status, and surgeon's preferences and abilities. Brubaker et al. [25] recommended LSC combined with the Burch surgery to prevent postoperative SUI and anterior vaginal wall prolapse. However, the consequence is that for every case of postoperative UI prevention, 6–11 cases of unnecessary anti-SUI surgeries may be required, which increases surgical trauma and risks. There is still some controversy regarding the combined treatment of surgical methods. Saida Abrar et al. [26] assessed the effect of POP and/or SUI on various domains of female sexual functions in patients before and after reconstructive surgery for these pelvic floor disorders. However, there have not been many reports on laparoscopic sacrocolpopexy and TVT-O on POP and SUI surgery, and there is a lack of follow-up and evaluation of postoperative quality of life of patients. Therefore, the innovation of this research is to review the clinical data of SUI patients complicated with POP treated by LSC and TVT-O to observe the clinical effect.

The article "Clinical Efficacy of LSC and TVT-O for Stress Urinary Incontinence Complicated with Pelvic Organ Prolapse and Factors Influencing Postoperative Urinary Function Recovery" was retracted in 2023. Reasons: suspected computer-generated content; unreliable results or conclusions; concerns about the data; concerns about the results or conclusions.

The results revealed notably longer OT and postoperative indwelling catheter time and higher IBL in the combination group versus the control group, while no distinct difference in anal exhaust time and postoperative LOS. As the surgical treatment performed in the combination group was LSC followed by TVT-O, the OT was longer with larger volume of blood loss, but the two arms showed no evident difference in postoperative recovery. Then, after observing the urodynamic indexes of the two groups, it was found that the initial bladder volume, maximum bladder volume, MFR, and average UF recovery time were markedly better in the control group. TVT-O is a tension-free vaginal tape that theoretically does not increase urethral resistance under unstressed conditions [27]. However, due to the compression of the sling on the periurethral tissue and the absence of tension standard of the sling as well as individual differences, postoperative uroschesis, urination difficulty, and decreased force of urination are easy to occur, affecting patients' postoperative recovery. Ek et al. [28] also believe that POP surgery combined with anti-UI surgery may result in decreased urinary flow rate, dysuria, uroschesis, and prolonged OT, rising the likelihood of developing perioperative complications. Our experimental results were verified by perioperative and urodynamic indicators. Subsequently, the observation of the long-term efficacy of the patients revealed that the ORR of the combination group was significantly higher, with better improved condition, QOL, and quality of sexual life. According to a British study [29], about 37–64% of women visit the gynecological urology department for sexual dysfunction. POP or SUI-induced sexual dysfunction usually includes sexual desire/arousal disorder, orgasmic disorder, and dyspareunia [30]. While studies reported sexual dysfunction problems in women with UI, some others focused on dyspareunia, low sexual desire, and colpoxerosis in POP patients [31]. Some research investigating the role of POP and/or anti-SUI surgery in female sexual function has shown that reconstructive operation for POP or SUI may not always restore optimum sexual function, but assuming no significant difference in sexual function after POP and/or SUI surgery, other research has pointed out that female sexual function is under the influence of POP and SUI and these pelvic floor diseases are significantly ameliorated postoperatively [32]. This research also shows that the combined surgical treatment can improve the patients' long-term QOL and sexual life treatment better, with a lower the incidence of complications. It may be due to that the puncture of medial obturator membrane during TVT-O operation and timely replacement of gloves after LSC effectively reduced vaginal traction, puncture injury, infection, and bladder wall injury, and improved pelvic floor function and bladder function, thus effectively reducing the risk of complications [33]. Finally, menopause, MFR, and preoperative RUV were analyzed as the influencing factors for normal urination. Studies have shown that [34, 35] good urethral function is closely related to the body's estrogen level and the blood supply of urethral mucosa. However, with the increase in age and the occurrence of menopause, female estrogen level reduces significantly, urethral blood supply decreases, urethral epithelium becomes thinner, and muscle atrophy occurs, which is not conducive to the recovery of micturition muscle function. The MFR is the maximum volume of urine discharged from the body through the urethra per unit time, which reflects the detrusor function [36]. Park et al. [37] comprehensively analyzed TVT-O, and the results showed that the maximum urine flow rate before and after surgery was 30.1 mL/s and 23.5 mL/s, respectively, with an average decrease of 6.6 mL/s. This suggested that the maximum urine flow rate is a useful estimate of the risk of voiding dysfunction and can predict the likelihood of postoperative urinary retention before surgery. If the MFR is low and urine discharge is limited, the UF recovery speed will be affected.

The article "Clinical Efficacy of LSC and TVT-O for Stress Urinary Incontinence Complicated with Pelvic Organ Prolapse and Factors Influencing Postoperative Urinary Function Recovery" was retracted in 2023. Reasons: suspected computer-generated content; unreliable results or conclusions; concerns about the data; concerns about the results or conclusions.

To sum up, for patients with SUI complicated with POP, LSC combined with TVT-O has better long-term efficacy and can significantly improve patients' QOL and achieve higher clinical effective rate, although the perioperative indicators are not prominent. Clinically, there is no consensus on whether the surgical treatment of SUI complicated with POP patients should be accompanied by anti-SUI surgery, and the results of this study offer a choice of surgical treatment in patients with SUI complicated with POP, which has certain clinical significance. This study analyzed the surgical value of SUI complicated with POP from the perspectives of surgical efficacy, postoperative functional recovery, and quality of life, providing some insight into clinical treatment decisions. Still, there is room for improvement in this research. Due to limited sample size, a large-scale, randomized, prospective, and multicenter systematic study is warranted to conduct comprehensive and long-term follow-up for evaluating the clinical value of the combined application of LSC and TVT-O. Our prospect is to provide a better surgical treatment plan for the needs of patients with POP combined with SUI, which can solve the needs of patients in one step, and provide more reference value for the clinical application of the combined application of the two surgical methods.

The article "Clinical Efficacy of LSC and TVT-O for Stress Urinary Incontinence Complicated with Pelvic Organ Prolapse and Factors Influencing Postoperative Urinary Function Recovery" was retracted in 2023. Reasons: suspected computer-generated content; unreliable results or conclusions; concerns about the data; concerns about the results or conclusions.

## Figures and Tables

**Figure 1:** Comparison of subjective evaluation indexes. (a) PFDI-20 score; (b) PIIQ-7 score; and (c) PISQ-12 score; ^*∗∗∗*^*P* < 0.001.

**Table 1:** General baseline data.

	Control group (*n* = 60)	Combination group (*n* = 65)	*χ* ^2^/*t*	*P*
Average age (years)	40.3 ± 5.1	40.1 ± 5.6	0.2082	0.8354
BMI (kg/m^2^)	23.8 ± 2.9	23.5 ± 2.6	0.6098	0.5431
Gravidity (times)	3.5 ± 1.5	3.3 ± 1.4	0.7711	0.4421
Parity (times)	2.1 ± 0.4	2.0 ± 0.3	1.5889	0.1146

*POP-Q*			0.4651	0.7925
II	15 (25.0)	18 (27.7)		
III	28 (46.7)	32 (49.2)		
IV	17 (28.3)	15 (23.1)		

*Ingelman-Sundberg classification*			1.2982	0.5226
Mild	16 (26.7)	20 (30.8)		
Moderate	30 (50.0)	35 (53.8)		
Severe	14 (23.3)	10 (15.4)		

*Pausimenia*			0.7813	0.3767
Yes	23 (38.3)	30 (46.2)		
No	37 (61.7)	35 (53.8)		

*Underlying diseases*				
Diabetes mellitus	8 (13.3)	11 (16.9)	0.3119	0.5765
Hypertension	9 (15.0)	14 (21.5)	0.8884	0.3459

**Table 2:** Comparison of perioperative indicators.

Groups	OT (min)	IBL (mL)	Postoperative indwelling catheter time (d)	Anal exhaust time (h)	Postoperative length of stay (d)
Control group (*n* = 60)	116.4 ± 27.4	97.6 ± 10.5	2.1 ± 0.5	34.8 ± 0.9	11.6 ± 3.2
Combination group (*n* = 65)	138.6 ± 31.8	105.6 ± 14.6	2.7 ± 0.3	35.1 ± 1.1	12.1 ± 3.8
*χ* ^2^/*t*	4.1653	3.4915	8.2073	1.6607	0.7921
*P*	**<0.0001**	**0.0006**	**<0.0001**	0.0993	0.4291

*Note.* Bold text means statistically significant.

**Table 3:** Comparison of urodynamic indexes.

Groups	Preoperative residual urine volume (mL)	Initial bladder volume (mL)	Maximum bladder volume (mL)	Maximum flow rate (mL/s)	Recovery time of urinary function		
					Average time (d)	≤3 d	>3 d
Control group (*n* = 60)	30.6 ± 6.8	301.6 ± 22.8	405.9 ± 34.3	27.1 ± 4.6	3.21 ± 0.46	23 (38.3)	37 (61.7)
Combination group (*n* = 65)	30.3 ± 7.3	272.6 ± 18.6	355.4 ± 31.8	23.4 ± 2.4	3.74 ± 0.71	13 (20.0)	52 (80.0)
*χ* ^2^/*t*	0.2372	7.8174	8.5419	5.6999	4.9905	5.1141	
*P*	0.8129	**<0.0001**	**<0.0001**	**<0.0001**	**<0.0001**	**0.0237**	

*Note.* Bold text means statistically significant.

**Table 4:** Comparison of POP-Q parameters.

		Control group (*n* = 60)	Combination group (*n* = 65)	*χ* ^2^/*t*	*P*
Aa (cm)	Before surgery	−2.2 ± 0.5	−2.1 ± 0.3	1.3679	0.1738
	6 months after surgery	−2.4 ± 0.3^*∗*^	−2.5 ± 0.4^*∗*^	1.5709	0.1187
Ba (cm)	Before surgery	−2.1 ± 1.1	−2.3 ± 1.0	1.0648	0.2890
	6 months after surgery	−2.5 ± 0.9^*∗*^	−2.6 ± 0.6^*∗*^	0.7361	0.4631
Ap (cm)	Before surgery	−2.8 ± 0.5	−2.7 ± 0.4	1.2392	0.2176
	6 months after surgery	−3.0 ± 0.8^*∗*^	−2.9 ± 0.7^*∗*^	0.7451	0.4576
Bp (cm)	Before surgery	−2.8 ± 1.0	−2.7 ± 1.1	0.5303	0.5968
	6 months after surgery	−3.1 ± 0.6^*∗*^	−3.0 ± 0.5^*∗*^	1.0151	0.3120
C (cm)	Before surgery	−4.5 ± 1.2	−4.4 ± 1.6	00.3927	0.6952
	6 months after surgery	−4.2 ± 1.1^*∗*^	−3.7 ± 1.3^*∗*^	2.3116	0.0225
D (cm)	Before surgery	−6.5 ± 1.8	−6.6 ± 2.0	0.2929	0.7700
	6 months after surgery	−5.5 ± 1.7^*∗*^	−3.9 ± 1.2^*∗*^	6.1157	**<0.0001**
TVL (cm)	Before surgery	5.3 ± 0.5	5.4 ± 0.4	1.2392	0.2176
	6 months after surgery	5.4 ± 0.2	7.0 ± 0.9^*∗*^	13.4633	**<0.0001**

*Note.* ^*∗*^ *P* < 0.05*vs* before surgery within the group; bold text means statistically significant.

The article "Clinical Efficacy of LSC and TVT-O for Stress Urinary Incontinence Complicated with Pelvic Organ Prolapse and Factors Influencing Postoperative Urinary Function Recovery" was retracted in 2023. Reasons: suspected computer-generated content; unreliable results or conclusions; concerns about the data; concerns about the results or conclusions.

**Table 5:** Comparison of objective response rate.

Groups	Cure rate	Improvement rate	Ineffective rate	Recurrent rate
Control group (*n* = 60)	35 (58.3)	15 (25.0)	6 (10.0)	4 (6.7)
Combination group (*n* = 65)	55 (84.6)	7 (10.8)	3 (4.6)	0 (0)
*χ* ^2^/*t*	10.6910	4.3571	1.3541	4.4771
*P*	**0.0011**	**0.0369**	0.2446	0.0344

*Note.* Bold text means statistically significant.

**Table 6:** Comparison of the incidence of complications.

Groups	Defecation discomfort	Infection	Dysuria	Bladder injury	Total incidence
Control group (*n* = 60)	2 (3.3)	3 (5.0)	3 (5.0)	3 (5.0)	11 (18.3)
Combination group (*n* = 65)	1 (1.5)	1 (1.5)	2 (3.1)	0 (0)	4 (6.1)
*χ* ^2^/*t*					4.3831
*P*					**0.0363**

*Note.* Bold text means statistically significant.

**Table 7:** Correlation of variables with recovery time of urinary function.

	≤3d (*n* = 36)	>3d (*n* = 89)	*χ* ^2^/*t*	*P*
*Age*			1.5351	0.2153
≤40	11 (30.6)	18 (20.2)		
>40	25 (69.4)	71 (79.8)		

*Menopause*			4.0531	**0.0441**
Yes	20 (55.6)	32 (35.9)		
No	16 (44.4)	57 (64.1)		

*Underlying diseases*			0.6339	0.4259
Yes	14 (38.9)	28 (31.5)		
No	22 (61.1)	61 (68.5)		

*Maximum flow rate*			5.0961	**0.0240**
≤24 mL/s	8 (22.2)	39 (43.8)		
>24 mL/s	28 (77.8)	50 (56.2)		

*Preoperative residual urine volume*			4.4001	**0.0359**
≤30 mL	22 (61.1)	36 (40.4)		
>30 mL	14 (38.9)	53 (59.6)		

*Note.* Bold text means statistically significant.

## Data Availability

The clinical data used to support the findings of this study are included within the article.
